The article "Hericium erinaceus mycelium and its isolated erinacine A protection from MPTP-induced neurotoxicity through the ER stress, triggering an apoptosis cascade" was retracted in 2021. Reasons: duplicated images; a conflict of interest.

# *Hericium erinaceus* mycelium and its isolated erinacine A protection from MPTP-induced neurotoxicity through the ER stress, triggering an apoptosis cascade

**DOI:** 10.1186/s12967-016-0831-y

**Published:** 2016-03-18

**Authors:** Hsing-Chun Kuo, Chien-Chang Lu, Chien-Heng Shen, Shui-Yi Tung, Meng Chiao Hsieh, Ko-Chao Lee, Li-Ya Lee, Chin-Chu Chen, Chih-Chuan Teng, Wen-Shih Huang, Te-Chuan Chen, Kam-Fai Lee

**Affiliations:** Department of Nursing, Chang Gung University of Science and Technology, Chiayi, Taiwan; Research Center for Industry of Human Ecology, Chang Gung University of Science and Technology, Taoyuan, Taiwan; Division of Colorectal Surgery, Department of Surgery, Chang Gung Memorial Hospital, Kaohsiung Medical Center, Chang Gung University College of Medicine, Kaohsiung, Taiwan; Department of Hepato-Gastroenterology, Chang Gung Memorial Hospital, Chiayi, Taiwan; Chang Gung University College of Medicine, Taoyuan, Taiwan; Division of Colon and Rectal Surgery, Department of Surgery, Chang Gung Memorial Hospital, Chiayi, Taiwan; Grape King Biotechnology Inc., Zhong-Li, Taiwan; Division of Nephrology, Kaohsiung Chang Gung Memorial Hospital and Chang Gung University College of Medicine, Kaohsiung, Taiwan; Department of Pathology, Chang Gung Memorial Hospital, Chiayi, Taiwan

**Keywords:** *Hericium erinaceus* mycelium, Erinacine A, Parkinson’s disease, Endoplasmic reticulum stress

## Abstract

**Background:**

*Hericium erinaceus* is an edible mushroom; its various pharmacological effects which have been investigated. This study aimed to demonstrate whether efficacy of oral administration of *H. erinaceus* mycelium (HEM) and its isolated diterpenoid derivative, erinacine A, can act as an anti-neuroinflammatory agent to bring about neuroprotection using an MPTP (1-methyl-4-phenyl-1,2,3,6-tetrahydropyridine) mouse model of Parkinson’s disease, which results in motor disturbances, in addition to elucidating the mechanisms involved.

**Methods:**

Mice were treated with and without HEM or erinacine A, after MPTP injection for brain injuries by the degeneration of dopaminergic nigrostriatal neurons. The efficacy of oral administration of HEM improved MPTP-induced loss of tyrosine hydroxylase positive neurons and brain impairment in the substantia nigra pars compacta as measured by brain histological examination.

**Results:**

Treatment with HEM reduced MPTP-induced dopaminergic cell loss, apoptotic cell death induced by oxidative stress, as well as the level of glutathione, nitrotyrosine and 4-hydroxy-2-nonenal (4-HNE). Furthermore, HEM reversed MPTP-associated motor deficits, as revealed by the analysis of rotarod assessment. Our results demonstrated that erinacine A decreases the impairment of MPP-induced neuronal cell cytotoxicity and apoptosis, which were accompanied by ER stress-sustained activation of the IRE1α/TRAF2, JNK1/2 and p38 MAPK pathways, the expression of C/EBP homologous protein (CHOP), IKB-β and NF-κB, as well as Fas and Bax.

The article "Hericium erinaceus mycelium and its isolated erinacine A protection from MPTP-induced neurotoxicity through the ER stress, triggering an apoptosis cascade" was retracted in 2021. Reasons: duplicated images; a conflict of interest.

**Conclusion:**

These physiological and brain histological changes provide HEM neuron-protective insights into the progression of Parkinson’s disease, and this protective effect seems to exist both in vivo and in vitro.

## Background

*Hericium erinaceus* (Lion’s mane or Yamabushitake) is an edible mushroom with medicinal properties; it grows on old or dead broadleaf trees. It is used as a food and herbal medicine in Japan and China without harmful effects [1]. The mushroom may be a good candidate for inducing neuronal differentiation and promoting neuronal survival [2]. Both the mycelium (erinacines A-I) and the fruiting bodies (Hericenone C-H) are the source of many bioactive extracts with drug efficacy. *Hericium erinaceus* has been extensively documented and possesses a range of therapeutic properties, such as antioxidant activity [3], hypolipidemic activity [4], hemagglutinating activity [5], antimicrobial activity [6], antiaging activity [7], immune modulation and anticancer activities [8, 9]. Erinacine A has small molecular weight components that are the major active agents isolated from the cultured mycelium of *H. erinaceus.* These diterpenoid compounds also play a role in varied functions, including neuroprotection through nerve growth factor (NGF) synthesis [10]. Therefore, *H. erinaceus* is attracting attention as a novel resource, not only for medicinal drugs, but also for dietary phytochemicals for disease prevention and health promotion through use of its biological properties [11]. Our previous study focused on exploring the biological agent of erinacine A from *H. erinaceus* mycelium and its structural elucidation by ethanol extraction and HPLC analysis techniques [12, 13]. However, the mechanism by which *H. erinaceus* mycelium and its isolated diterpenoid derivative, erinacine A, promote neuron cell survival and protection from MPTP-induced neurotoxicity remains poorly understood, as does the mechanism by which *H. erinaceus* mycelium and erinacine A initiate neuroprotection against MPTP injury to the brain.

Parkinson’s disease (PD) involves a distinct sequence of events behind the selective neuronal death that occurs in PD, but these events are not fully understood [14–16]. Numerous diseases of the nervous system, such as Parkinson’s disease (PD) produce excessive free radical generation (reactive oxygen species [ROS] and reactive nitrogen species [RNS]), which then cause oxidative damage. These include lipids, oxidative S-nitrosylation proteins and nucleic acids, which have been linked to apoptosis by the high levels of ROS in dopamine neurons due to dopamine metabolism. Various disease models for PD also show the involvement of the drug 1-methyl 4-phenyl 1,2,3,6-tetrahydropyridine (MPTP) [17, 18]. Furthermore, the MPTP animal model is useful for the study of neurodegeneration in PD. The neurotoxic effects of MPTP are thought to be mediated by its metabolite 1-methyl-4-phenylpyridinium ion (MPP+) and monoamine oxidase-B (MAO-B) in neuron cells, leading to a number of deleterious effects on cellular function, such as impairing the dopaminergic nigrostriatal neurons, generating free radicals from the mitochondria and a neuroinflammatory response, similar to those seen in PD [19, 20]. Our previous investigation focused on exploring the biological agent of erinacine A from *H. erinaceus* mycelium, its structural elucidation by ethanol extraction and HPLC analysis techniques [12, 13]. However, the mechanism by which *H. erinaceus* mycelium and its isolated diterpenoid derivative, erinacine A, are able to effectively improve the neuroprotective effects of the endoplasmic reticulum (ER) stress pathway and apoptosis, as well as how the signal cascades become activated, remain poorly understood.

The article "Hericium erinaceus mycelium and its isolated erinacine A protection from MPTP-induced neurotoxicity through the ER stress, triggering an apoptosis cascade" was retracted in 2021. Reasons: duplicated images; a conflict of interest.

Numerous studies have demonstrated that the ER stress pathway might be crucial in various CNS degenerative diseases [21]. In fact, ER stress may be related to neuronal death. In particular, the JNK/p38 MAPK/CHOP pathways involved in ER-stress-induced apoptosis in the neurons are implicated in PD [22]. In addition, energy metabolism with cultured neuronal cells, including dopaminergic neurons, showed that MPP + triggers ER stress and induces a number of genes [23]. Thus, extreme oxidant and peroxide levels from the neurotoxicity of MPTP suggest that inhibition of antioxidant defenses results in inflammatory effects and generation of ROS or RNS found in PD-related neuron damage [24, 25]. MPTP injury of the brain then induces oxidative stress, which leads to activate the multiple-cellular-signaling pathway, such as the IRE1α pathway. IRE1α binds TNF receptor-associated factor 2 (TRAF2), apoptosis signal-regulating kinase 1 (ASK1) and downstream kinases that further activate Jun N-terminal kinase (JNK) and nuclear factor-κB (NF-κB), which has also been linked to PD [26, 27]. In the present study, we explore the biological agent of *H. erinaceus* mycelium that is associated with protection against ER stress and loss of dopaminergic nigrostriatal neurons.

In our previous study, we investigated the molecular mechanisms underlying *H. erinaceus* that inhibit global cerebral ischemic injury via inactivation of the iNOS/RNS and p38 MAPK/CHOP pathways, which may be among the possible pathways involved in stroke-related neuron injury [12, 13]. In the present study, we assess the neuroprotective effect of *H. erinaceus* mycelium and its isolated compound erinacine A, as well as its relevance to idiopathic PD in the MPTP mouse model. We were able to demonstrate that *H. erinaceus* mycelium, a known antioxidant, is able to protect against the endoplasmic reticulum stress induced by the loss of dopaminergic neurons and disordered motor function by MPTP injury. This results in its isolated compound erinacine A promoting neuronal cell survival due to MPP+ -mediated induction expression of Fas and Bax via IRE1α/TRAF2 complex formation and phosphorylation of the JNK1/2, p38 and NF-kB pathways. Moreover, developing more effective dietary *H. erinaceus* mycelium for PD is an important goal.

The article "Hericium erinaceus mycelium and its isolated erinacine A protection from MPTP-induced neurotoxicity through the ER stress, triggering an apoptosis cascade" was retracted in 2021. Reasons: duplicated images; a conflict of interest.

## Methods

### *Hericium erinaceus* extracts and analysis of erinacine A

Fresh mycelium of *H. erinaceus* was extracted with ethanol. The extract was concentrated and fractionated by solvent partition between ethylacetate and water. The ethylacetate fraction was subjected to silica gel column chromatography using *n*-Hexane–ethylacetate as the eluent. The Hexane–acetone eluate was subjected to silica gel column chromatography according to the previous study [9, 12, 13]; HPLC analysis of erinacine A was executed according to the previous study with minor modifications. The analytical column used was a COSMOSIL 5C18-AR-II (250 × 4.6 mm; particle size 5 μm, Nacalai USA, Inc., Kyoto, Japan). Separation was performed at 40 °C using two different gradients for the mobile phase, which consisted of two solvents, methanol (A) and 2.0 % acetic acid in water (B). The gradient elution had the following profile: 0–20 min, 60–90 % (A); 20–25 min, 90 % (A). The retention time of erinacine A was approximately ~17 min at a flow rate of 1.0 mL/min with a scanning UV wavelength at 340 nm. The 3 mg/g erinacine A in the *H. erinaceus* extracted with 85 % ethanol was confirmed and quantified by HPLC as shown in Fig. 1 [12, 13]. Chemical compounds studied in this article Erinacine A (PubChem CID: 10410568).

**Fig. 1:** Simplistic flow chart of neuroprotective activities of *Hericium erinaceus* mycelium (*HEM*) in a MPTP treated animal model

### Animals

C57BL/6 mice (8–10 weeks old, 20–28 g) were kept individually in a 12-h light/dark cycle cage and had free access to water and food. Animal care and the general protocols for animal use were approved by the Institutional Animal Care and Use Committee of Chang Gung University of Science and Technology. Mice were operated on according to the modified MPTP-induced PD’s model, can be induced by the intraperitoneal injections of MPTP-HCl (30 mg/kg; Sigma, St. Louis, MO) or saline in 5 day. Four groups (six mice in each group) were randomly assigned to a sham control group, a MPTP group, three *H. erinaceus* wet mycelia (HEM) groups (5.38, 10.76 and 21.52 mg) and erinacine A groups (1 mg/kg). HEM was dissolved in water (H_2_O) and mice received HEM oral administration indicated during the 25 days before the onset of MPTP induction and HEM starting after the first MPTP injection and continuing through 5 additional days. Erinacine A was dissolved in dimethyl sulfoxide (DMSO) and administered intraperitoneally for 5 days before the MPTP induction. The sham-operated group animals received an equivalent volume of saline. Mice were killed 5 days after MPTP injection and brains were harvested, sectioned, and processed [28].

The article "Hericium erinaceus mycelium and its isolated erinacine A protection from MPTP-induced neurotoxicity through the ER stress, triggering an apoptosis cascade" was retracted in 2021. Reasons: duplicated images; a conflict of interest.

### Chemical reagents and antibodies

Mouse monoclonal antibodies against tyrosine phospho-Hydroxylase (Ser31), GAPDH, β-actin, 4-Hydroxy-2-nonenal (4-HNE), Nitro-tyrosine, CHOP, Fas, Bax, NFkB p65, Histone H1, TRAF2, IRE1α, and phospho-IKB-β were purchased from Santa Cruz Biotechnology (Santa Cruz, CA, USA). Rabbit monoclonal antibodies against phospho-p38 MAPK (Thr180/Tyr182) and phospho-JNK1/2 (Thr183/Tyr185) were purchased from Cell Signaling Technology (Beverly, MA, USA). The TdT-mediated dUTP Nick End Labeling (TUNEL) kits were purchased from Roche (Germany). MPP+ (1-methyl-4-phenylpyridinium), SDS, NP-40, while sodium deoxycholate, protease inhibitor cocktail was purchased from Sigma (St. Louis, MO, USA).

### Behavioral testing

Behavioral assessments on mice were made 1–6 days after MPTP injection. Motor performance was assessed with a rotary rod apparatus using a protocol similar to that described [29]. For the rotarod tests, the paradigms were used: rocking—direction of rotation with each full turn of the rod at 10 rpm for 3 min to a level just below the bottom of the rod. The mice were placed on the rotating rod and the time until they fell off was recorded. This was repeated six times until the total time on the rod for the control group was 3 min. Both the total time spent on the rotating rod for each mice, five groups (Control, MPTP, HEM), were recorded.

### Immunohistochemistry

After the administration of a large dose of chloral hydrate, the mice were killed by decapitation 8 days after MPTP treatment. The brains were quickly removed and placed in ice-cold saline for 10 min. Next, the brains were cut into seven 4 μm-thickness slides transversely from neuron impairment area using a mouse brain matrix (Harvard Apparatus, MA, USA) and then immediately fixed in 10 % formalin overnight. The brain sections were then dehydrated with graded ethanol, passed through chloroform, and embedded in paraffin, which were assessed by hematoxylin and eosin (H and E) staining. Paraffin sections of the striatum and substantia nigra were used for immunohistochemistry (IHC). Staining was performed using a biotinylated secondary antibody (Vectastain Universal Elite ABC Kit). Monoclonal rabbit antibodies against tyrosine Hydroxylase, nitro-tyrosine, 4-HNE and Fas (CD95) were diluted in a ratio of 1:100. The omission of primary antibodies was used as the negative control. Using the slides, the presence of cytoplasm stained with brown was scored as positive. The protein expression were quantitatively evaluated using an Olympus Cx31 microscope with an Image-pro Plus medical image analysis system. The digital images were captured using a digital camera (Canon A640). The positive area and optical density of the positive cells were determined by measuring three randomly selected microscopic fields (100×, 200× magnification) on each slide. The IHC index was defined as average integral optical density (AIOD) (AIOD = positive area × optical density/total area) [30].

The article "Hericium erinaceus mycelium and its isolated erinacine A protection from MPTP-induced neurotoxicity through the ER stress, triggering an apoptosis cascade" was retracted in 2021. Reasons: duplicated images; a conflict of interest.

### Cell culture

The mouse N2a (Neuro-2a) cells were purchased from the American Tissue Culture Collection (ATCC, USA). Cells were grown in Dulbecco’s Modified Eagle Medium (DMEM) (Gibco) supplemented with 10 % fetal calf serum (Gibco), non-essential amino acids, 1 mM sodium pyruvate and 1 % antibiotics (100 units/mL of penicillin and 100 μg/mL of streptomycin). All experiments were performed in plastic tissue culture flasks, dishes or in microplates (Nunc, Naperville, Denmark). Incubation was carried out at 37 °C in a humidified atmosphere of 5 % CO2 and 95 % air [31].

### Assessment of cell viability and apoptosis assay

Cell viability, as previously reported by MTT quantitative colorimetric assay, was capable of detecting viable cells. The cells were seeded at 2 × 10^4^ cells/ml density and incubated with MPP + for 24 h. Thereafter the medium was changed and incubated with MTT (0.5 mg/ml) for 4 h. The viable cell number is directly proportional to the production of formazan following solubilization with isopropanol, which can be measured spectrophotometrically at 563 nm [31]. Annexin V/propidium iodide (Biosource International, USA) was used to quantify the percentage of apoptosis cells. Flow cytometric analysis was performed with a FACSCaliber using CellQuest software. Data were analyzed with CellQuest and WinMDI software. The apoptotic cells (V+/PI-) were measured by the fluorescence-activated cell sorter analysis in a FACS analyzer (Becton–Dickinson). The data represented three independent experiments [32].

The article "Hericium erinaceus mycelium and its isolated erinacine A protection from MPTP-induced neurotoxicity through the ER stress, triggering an apoptosis cascade" was retracted in 2021. Reasons: duplicated images; a conflict of interest.

### Preparation of total cell extracts and immunoblotting analysis

Cells were lysed with a buffer containing 1 % NP-40, 0.5 % sodium deoxycholate, 0.1 % sodium dodecyl sulfate (SDS) and a protease inhibitor mixture (phenylmethylsulfonyl fluoride, aprotinin and sodium orthovanadate). The total cell lysate (50 μg of protein) was separated by SDS–polyacrylamide gel electrophoresis (PAGE) (12 % running, 4 % stacking) and analyzed by using the designated antibodies and the Western-Light chemiluminescent detection system (Bio-Rad, Hercules, CA), as previously described [31].

### Statistical analyses

Data were reported as the mean ± standard deviation (SD) of three independent experiments and were analyzed by one-way analysis of variance (ANOVA). The data were analyzed using the SAS software statistical package “SigmaPlot,” version 9.0 (SAS Institute Inc., Cary, NC, USA) [33].

## Results

### *Hericium erinaceus* mycelium (HEM) inhibits the cytotoxic effect of neuron cells in the MPTP-treatment animal model

Our previous study demonstrated that *H. erinaceus* mycelium and its structural analog erinacine A have nerve-growth properties, allowing them to aid in the prevention of ischemic injury to neurons in the central nervous system of excessive oxidative stress subjects [12, 13]. Based on these studies, we assayed whether *H. erinaceus* mycelium provides substantial therapeutic advantages by suppressing brain impairment in a mouse model that resembles PD. Figure 1 shows the neuroprotection of HEM in an MPTP-treated animal model. Figure 2 shows the expressions of the results of TUNEL as well as tyrosine hydroxylase (dopaminergic neurons). There was also a reduction in the number of positive TUNEL cells in the striatum and substantia nigra, a marker of apoptosis, when the MPTP mice treated with HEM were compared with the untreated MPTP mice (MPTP = 38 ± 5; 10.76 and 21.52 mg/day, HEM = 24 ± 3 and 7 ± 2, * <0.05). Tyrosine hydroxylase (TH) is expressed exclusively in most dopaminergic neuronal cell types. TH is the enzyme responsible for the conversion of the amino acid l-tyrosine to dopamine, while PD can be indicated as a TH-deficiency syndrome of the striatum. Immunoreactivity of phospho-Tyrosine hydroxylase was found to reside mostly in the brain striatum area in the MPTP group 24 h after administering HEM. Quantification of the dopaminergic neuron cells in terms of pathology showed that the dosage of MPTP administration was inclined to decrease the number of normal neurons compared to the control group. However, a significant increase was found between the MPTP and MPTP + HEM (10.76 and 21.52 mg/day) group (untreated MPTP = 32 ± 5; HEM treated MPTP = 72 ± 6 *#* <0.05 and 116 ± 13) (see Fig. 2c).

The article "Hericium erinaceus mycelium and its isolated erinacine A protection from MPTP-induced neurotoxicity through the ER stress, triggering an apoptosis cascade" was retracted in 2021. Reasons: duplicated images; a conflict of interest.

**Fig. 2:** Effect of *Hericium erinaceus* mycelium (HEM) on brain histological examination in MPTP treated animal model. MPTP animal models (MPTP injection and brains harvested) were performed on mice described in “Methods” section. **a** Histological examination of brain were revealed to striatum and substantia nigra zones as indicated by immunohistochemical staining of TUNEL. Representative brain sections stained as saline infusion control group (*I*); Mice with MPTP injection (*II*); HEM treatment (10.76 and 21.52 mg/day) (*III*, *IV*); Apoptotic cells were measured under microscopy as described in “Methods” section. The MPTP group exhibited dopamine deficiency syndrome of the striatum, as indicated by apoptotic cells (*filled arrow*). Magnification, ×100. **b** Histological examination of brain were revealed in brain, as indicated by immunohistochemical staining of tyrosine Hydroxylase p-Ser 31. Magnification, ×200. The cells were counted from 10 fields (200× magification) of each brain sample. **c** The results from statistical analysis are the means of cells and were calculated per microscope field from six animals per group. Data are expressed as mean ± SD of independent experiments. *p < 0.05, MPTP group versus MPTP + HEM group. ^#^ *P* < 0.05, MPTP group versus MPTP + HEM group

### HEM treatment-attenuated brain protein ROS oxidants and behavioral impairment in mice with MPTP intoxication

In a previous study, an animal model of Parkinson’s disease showed the result of the presence of excessive free radicals after brain tissue damage; these have been reported to damage dopamine neurons due to dopamine formation for PD [23]. These findings demonstrated that HEM was able to inhibit oxidative nitrotyrosine proteins and lipid peroxidation 4-HNE, resulting in the dopaminergic nigrostriatal neurons’ apoptosis. This suggests that the ER stress effectors of CHOP via p38 MAPK may contribute to the neuroprotective effects by MPTP administration (Fig. 3, *p* < 0.05). Figure 4 shows the neuroprotective activities of HEM in an MPTP-treated animal model. Motor function of MPTP injection of HEM was also determined by a rotary rod apparatus, in comparison to an MPTP group. Five days after MPTP treatment, the mice showed significant motor function, as indicated by a decrease in the time periods on a rotary rod at 6 days, as compared to the control group MPTP mice (*p* < 0.05, n = 6). Significant differences were found between the HEM-treated and MPTP groups. The HEM group showed reduced motor dysfunction in a dose-dependent manner compared to the MPTP group (*p* < 0.01, n = 6; Fig. 3). Based on these studies, we tested whether HEM administration provided a protection of oxidative stress on densitometric analysis of neurotrophic factors in the brain striatum. As shown in Table 1, infusion of MPTP had a pro-inflammatory effect on brain injury, as shown through enzymatic analyses of the MPTP treatment group compared to a healthy control group. Dopamine, NGF and glutathione (GSH) levels were significantly lowered in the MPTP treatment group (MPTP infusion vs. normal saline infusion, *p* < 0.05, n = 6). Neuron GSH levels have recently been established as an indicator of oxidative stress in various diseases. The administration of the HEM groups significantly (HEM treatment vs. MPTP infusion, * <0.01, n = 6) elevated dopamine, NGF and the GSH level in the MPTP group.

The article "Hericium erinaceus mycelium and its isolated erinacine A protection from MPTP-induced neurotoxicity through the ER stress, triggering an apoptosis cascade" was retracted in 2021. Reasons: duplicated images; a conflict of interest.

**Fig. 3:** Effect of *Hericium erinaceus* mycelium (*HEM*) on brain histological nitrotyrosine and 4-HNE protein expression in MPTP animal model. Histological examination of brain were revealed to somata of dopamine neurons by immunohistochemical staining. **a** Mice were sacrificed and the brains were separated. Representative brain sections stained control group (*I*); Mice treated with MPTP at 6 days (*I*); HEM administration [10.76 (*III*) and 21.52 (*IV*) mg/day] staining of nitrotyrosine (**a**) and 4-HNE (**b**) protein in brain tissue. **c** Evaluation of nuclear protein expression and nitrotyrosine and 4-HNE expression were quantitative in the striatum. The area of dopamine neurons positive stained area from the SN was evaluated from three randomly selected observation fields of each brain section. Quantitative of immunohistochemical proteins by average integrated optical density (*AIOD*). Positive stained area was evaluated from three randomly selected observation fields of each liver section. Data were expressed as mean ± SD (n = 6/group). *p < 0.05, nitrotyrosine expression, MPTP group versus MPTP + HEM group.^ #^ *P* < 0.05, 4-HNE expression, MPTP group versus MPTP + HEM group

**Fig. 4:** Effect of *Hericium erinaceus* mycelium (*HEM*) treatment on motor function by the rocking rotarod assessment of coordination. Mean duration (in seconds) of the time spent on the rocking rotarod as a function of increasing motor function for MPTP and HEM administration mice. At 5 days after the MPTP injection, the mice exhibited a significant motor dysfunction as indicated by a decrease in the time period on rotarod. The mice with MPTP treated with HEM(III) and assessed by rotarod apparatus. Data were expressed as mean ± SD (n = 6/group). *p < 0.05, 4 days, control group versus MPTP and MPTP + HEM groups.^ #^ *P* < 0.05, 5 days, MPTP group versus MPTP + HEM groups. & *P* < 0.05, 5 days, MPTP group versus MPTP + HEM groups

**Table 1:** Biochemical effects of MPTP administration animal model by *Hericium erinaceus* mycelium

Neurotoxic effects of the striatum					
	Control (n = 6)	MPTP (n = 6)	MPTP + HEM 5.38 mg/day (n = 6)	MPTP + HEM 10.76 mg/day (n = 6)	MPTP + HEM 21.52 mg/day (n = 6)
Dopamine (ng/ml)	3.6 ± 0.15	1.7 ± 0.1	3.1 ± 0.1*	3.8 ± 0.1*	4.1 ± 0.1*
NGF (ng/ml)	2.8 ± 0.5	1.2 ± 0.1	1.9 ± 0.3*	2.3 ± 0.4*	2.7 ± 0.3*
GSH/mg	140 ± 11	62 ± 6	94 ± 8	134 ± 10	138 ± 8*

* *P* < 0.05, when compared with MPTP group

The article "Hericium erinaceus mycelium and its isolated erinacine A protection from MPTP-induced neurotoxicity through the ER stress, triggering an apoptosis cascade" was retracted in 2021. Reasons: duplicated images; a conflict of interest.

### Inhibition effects of erinacine A treatment on MPP + -induced ROS-related apoptosis and the ER stress-signaling mechanisms

Our previous findings demonstrated the effects of the biological agent of erinacine A from HEM fractionation and its effect on ischemia reperfusion injury. This suggests that the inactivation of the iNOS/RNS and p38 MAPK/CHOP pathways may contribute to the neuroprotective effects for both cortical and subcortical infarctions. MPTP exerts its neurotoxic effect through biological activation by MPP+, leading to mitochondrial energy loss, generation of toxic ROS and neuron cell death [34]. To clarify whether erinacine A has an inhibitory effect on the MPP+ model of neuronal injury that is cytotoxic to N2a cells and the molecular mechanisms underlying the MPP+ -mediated activation of IRE1a-inducing Jun N-terminal kinase (JNK1/2) and p38 MAP Kinase (MAPK), we induced N2a cells to MPP+ for 24 h, performed MTT assays and examined the protein levels of the ER stress-signaling pathway. Significantly decreased cell death was found in the erinacine A group compared to the MPP+ group (Fig. 5a). As shown in Fig. 5b, the extent of apoptosis of MPP+ induction was quantified as a percentage of annexin V-positive cells and shown as 20 %. Erinacine A treatment of N2a cells also resulted in increased neuron survival by 6 and 3 %, respectively. Erinacine A might have neuroprotection effects on neuron injury caused by oxidative stress of MPP+.

**Fig. 5:** Effect of MPTP on assessment of cell viability in N2a cells for 24 h. **a** after 24 h their viability was measured using an MTT assay. **b** After an indicated treatment for 24 h, the cells were stained with FITC-conjugated Annexin-V and PI for flow cytometry analysis as described in “Methods” section. The percentages presented in each frame depicted the apoptotic cells. *p < 0.05, indicates significant difference compared to an untreated group of N2a

### Erinacine A prevented cell death and was involved in the modulation of IRE1α/ΤRΑF2 complex levels, as well as ER-associated protein expression by MPP+ in neuron cells

Our results clearly showed that MPP+ resulted in neuron cell death and that oxidative damage was relative to the expression of Fas, Bax and CHOP, as well as to activation of the ER stress-signaling pathway, such as the p-JNK1/2, p38 MAPK and NF-κB triggering pathways, which may function downstream of the ER stress to induce apoptosis in response to neuronal damage, as an index of excessive oxidative damage with Western blotting (Fig. 6a). Conversely, treatment with erinacine A also resulted in a significant inhibition of JNK1/2 and p38 phosphorylation and ER-associated protein expression for 24 h. In addition, erinacine A was also found to induce effects on the IRE1α/ΤRΑF2 association (Fig. 6). In order to verify the effects of oral administration of HEM and erinacine A on the relationships between neuroprotection, inflammation and ER stress in the brain, Fas protein was selected for further examination using immunohistochemistry assays in vivo after MPTP injury and HEM treatment. As shown in Fig. 7, mice with MPTP impairment demonstrated increased expression of Fas (CD95) in the brain tissue samples. In particular, HEM and relative erinacine A treatment resulted in a significant reduction of Fas expression. These results are consistent with the results in vitro, indicating that HEM is applicable when protecting MPTP-induced brain neuron injury. Taken together, the results and the data showed that *H. erinaceus* mycelium and relative erinacine A administration in neuron cells is essential to involvement in oxidative stress-signaling MPP+ -mediated cell death along both IRE1α and JNK1/2/NF-κB-related pathways.

The article "Hericium erinaceus mycelium and its isolated erinacine A protection from MPTP-induced neurotoxicity through the ER stress, triggering an apoptosis cascade" was retracted in 2021. Reasons: duplicated images; a conflict of interest.

**Fig. 6:** Erinacine A mediated and ER-associated proteins expression between untreated (control) and treated (MPP+) in N2a cells. **a** Nuclear and whole cell lysate proteins were prepared and analyzed by Immunoblotting, using antisera to detect Fas, Bax, p-JNK, p-p38,CHOP, NF-kB p65, p-IKB-b and IRE1a (b-actin and Histone H1 served as the internal control). The association of TRAF2 with IRE1-a was determined by immunoprecipitation with TRAF2 followed by western blot with anti-IRE1-a antibody. **b** Protein levels were quantified by densitometric analysis with the control being set at 100 %. Data presented in western blot are derived from a representative study, and comparisons of protein expression are calculated from three independent experiments. *P < 0.05, when compared with control untreated group

**Fig. 7:** Effect of *Hericium erinaceus* mycelium (*HEM*) on brain histological Fas protein expression in MPTP treated animal model. Histological examination of brain were revealed to striatum and substantia nigra zones as indicated by immunohistochemical staining. Representative brain sections stained as saline infusion control group (*I*); Mice with MPTP injection (*II*); HEM treatment (5.38, 10.76 and 21.52 mg/day) (*III*, *IV*, *V*); Erinacine A (i.p. *VI*); The results from statistical analysis are the means of cells and were calculated per microscope field from six animals per group. Data are expressed as mean ± SD of independent experiments. *p < 0.05, MPTP group versus MPTP + HEM group and MPTP + EA group

The article "Hericium erinaceus mycelium and its isolated erinacine A protection from MPTP-induced neurotoxicity through the ER stress, triggering an apoptosis cascade" was retracted in 2021. Reasons: duplicated images; a conflict of interest.

## Discussion

ER stress-induced apoptosis is implicated in various pathological conditions, but the mechanisms of *H. erinaceus* mycelium on the suppression of oxidative stress and JNK/p38 MAPK as well as Fas, Bax and CHOP protein expression, which confer neuroprotection in PD involving ER stress–mediated signaling to neuron apoptotic pathways, remain unclear. It has been previously reported that a number of *H. erinaceus* extracts, used as a medicinal mushroom, can improve sleep quality, ameliorate depression and neurodegenerative disease, and improve cognitive impairment [35]. Moreover, it was reported that polysaccharides purified from the liquid culture broth of HEM and erinacine A enhanced the growth of mice adrenal nerve cells, improved the extension of neurite extension and expanded catecholamine in the brain of mice. Recently, studies were conducted on the synergistic effects of HEM extracts and exogenous NGF on neurite outgrowth in a glioma cell line. These studies demonstrate that the HEM extracts contain certain neuroactive components that induce NGF synthesis and promote neurite outgrowth, which has been shown to be a mycelium- growth-associated metabolite that stimulates NGF synthesis in cultured astrocytes [7]. Using an in vivo MPTP animal model and mouse neuron cell culture MPP+ -induced apoptosis (Fig. 1), our in vivo data demonstrated that the dopaminergic lesions and oxidative stress in the striatum and substantia nigra, as well as motor disorder, were significantly decreased after treatment with HEM (Figs. 2, 3, 4). In addition, we deployed several neuron cell death assays to confirm that the MPP+ damage, as measured by brain neuron death, is significantly decreased with erinacine A treatment at the concentration of 5 μM for 24 h in N2a cells (Fig. 5).

Studies have shown that ER stress- and inflammation-induced apoptosis is a key pathogenic event in disease processes as divergent as metabolism disease, cancer, hepatitis, heart disease and neurological diseases [5, 8, 22, 36]. The overall objective of this study made it necessary to develop more effective drugs from natural compounds of edible mushrooms to prevent neuronal death at high MPP+ exposures related to the mechanism of ER stress-induced apoptosis. The specific goal was linking upstream ER stress-mediated events to downstream apoptosis execution pathways in a model involving the JNK1/2, p38, NF-kB and CHOP pathways. Of current interest is the concept that prolonged CHOP expression leads to the release of ER calcium stores resulting from ER stress-induced expression of the Fas death receptor and Bax mitochondrial pathways of apoptosis through a pathway involving JNK and p38. Figure 6 shows that treatment of N2a cells with erinacine A increased the level of phosphorylated JNK and p38 MAPK as a result of an upregulation of CHOP and NFκB at 24 h, as well as a decrease in the Fas/Bax expression and IRE1α/TRAF2 complex interaction as early as 3 h. Our results showed that erinacine A inhibited MPP+ -induced neuron damage by inactivating oxidative stress-dependent CHOP expression. We also showed that both the Fas and Bax pathways, through induction of the Fas receptor itself and the mitochondrial pathway by MPP+ , and then specifically erinacine A, reduced the production of the ER stress-signaling pathway in dose-relative inhibition. Moreover, our histopathological and immunohistochemical assays provide unique evidence suggesting that HEM is able to suppress neuron impairment in MPTP mice at doses below the safe starting-dose range (Conversion of Animal Doses), and that this involves the significant inhibition of neuron death and Fas expression (Fig. 5). These findings provide an integrated, unique mechanism linking the ER stress to apoptosis, and suggest that it is feasible to determine whether *H. erinaceus* and relative erinacine A are able to effectively improve the neuroprotective effects for intervention directed against PD’s ER stress-induced apoptosis.

The article "Hericium erinaceus mycelium and its isolated erinacine A protection from MPTP-induced neurotoxicity through the ER stress, triggering an apoptosis cascade" was retracted in 2021. Reasons: duplicated images; a conflict of interest.

Studies have shown that natural phytochemicals from certain plants have the capability to exert neuroprotective effects in various experimental models of neurological disorders, and also to have cytotoxic effects on cancer cells [13, 37]. Furthermore, reducing oxidative stress-induced free radicals via an antioxidant effect has been shown to protect against the neuronal damage caused by neurotrophin deficiencies and toxin-induced degenerative diseases in response to chemopreventive drugs, such as dietary phytochemicals, phenols, alkaloids, flavonoids and mushrooms [38]. Moreover, finding a suitable neuroprotective agent is needed since this is a very important property with regard to its ability to cross the blood–brain barrier (BBB). To validate these findings, further study of *H. erinaceus* is needed to determine whether there are mediated actions to reach the target sites of the CNS in mice. However, phytochemicals that regulate neurodegenerative disease by targeting neurotrophins might provide a promising future. Both NGF and BDNF are expressed in dopaminergic neurons, suggesting that these act as a survival factor for the trophic support of neurons. Phytochemicals that potentiate neurotrophins and activate Trk receptors may serve to prohibit the onset of neurodegenerative PD [39]. On the other hand, it has been shown that JNK and p38 MAPK stress protein kinases are involved in inflammation and oxidative stress in neurodegenerative neuronal death in PD [36]. Our results showed that the upregulation of NGF protein and dopamine affected the striatum neuron cell with an increase of the antioxidative indicator GSH; these resulted in inhibitors targeting JNK and p38MAPK, preceded by the administration of *H. erinaceus* mycelium (Table 1; Fig. 6).

## Conclusion

In this study, we evaluated the molecular mechanisms underlying the roles of *H. erinaceus* against MPTP-induced neurotoxicity. Consequently, based on MPTP-treated mice, our results imply the possibility of a toxic effect of MPTP, a food provided by the mushroom components of *H. erinaceus*, on N2a cells and enable the evaluation of the protective ability and the underlying mechanisms against MPP+ cytotoxicity. In vivo study demonstrated that *H. erinaceus* mycelium decreased the brain dopamine neuronal loss and motor function. Our study showed that erinacine A inhibited the neuron cell apoptosis as a result of oxidative stress signaling and the JNK/p38/NF-κB/CHOP/Fas/Bax pathways (Fig. 8). These results provide insights into the neuroprotective activity of erinacine A of the *Hericium erinaceus* mycelium, which thus may be promising candidates for the treatment of neurodegenerative diseases such as PD.

**Fig. 8:** Schematic presentation of the ER Stress-signaling pathways involved in *Hericium erinaceus* mycelium and erinacine A suppressed MPP-induced apoptosis in N2a cells. *Hericium erinaceus* mycelium has neuroprotective potential through blocking oxidative stress MPTP-induced neuron damage and that erinacine A contribute to the protective action. The inhibition of effect of MPP on the ER stress triggering production of ROS activates IRE1a/TRAF2 complex formation and phosphorylation of JNK1/2, p38 and NF-kB pathways, which inhibits the Fas and Bax up-regulation and decreases an apoptosis cascade
